# Current Research on Complementary and Alternative Medicine in the Treatment of Premature Ovarian Failure: An Update Review

**DOI:** 10.1155/2022/2574438

**Published:** 2022-06-23

**Authors:** Yue Li, Meng-Yu Yan, Qiao-Chu Chen, Ya-Ya Xie, Chen-Yu Li, Feng-Juan Han

**Affiliations:** ^1^Heilongjiang University of Chinese Medicine, Harbin 150040, China; ^2^Department of Obstetrics and Gynecology, The First Affiliated Hospital of Heilongjiang University of Chinese Medicine, Harbin 150040, China

## Abstract

Complementary and alternative medicine (CAM) encompasses a wide range of different non-mainstream therapies that have been increasingly used for the treatment or adjunct treatment of various ailments, with premature ovarian failure (POF) being one of the most common conditions treated with CAM. This review updates the progress of CAM in the treatment of POF, and we focus specifically on reviewing the evidence for the efficacy and mechanisms of a range of CAM treatments in POF, including single herbal medicines and their active ingredients, compound Chinese medicines, acupuncture and moxibustion, psychotherapy, exercise, vitamins, massage, and dietary supplements. According to the literature, CAM is very helpful for improving POF symptoms, and we hope to provide some instructive suggestions for clinical treatment and experimental research in the future. However, more clinical trials are needed to prove the safety of CAM.

## 1. Introduction

Premature ovarian failure (POF) is a common endocrine disease leading to female amenorrhea and infertility. It is characterized by high expression of gonadotropin (follicle-stimulating hormone (FSH) ≥ 40 mIU/ml), low expression of estradiol (E2), and poor follicular development in women under 40 years old. Clinical symptoms are also accompanied by perimenopausal symptoms such as hot flashes, sweating, mood swings, sleep disorders, and low sexual desire [1–3]. At present, it is considered that the occurrence and development of POF are closely related to gonadotropin-related disorders [4], immune factors [5, 6], infectious factors [7, 8], iatrogenic factors [9], lack of metabolism-related enzymes [10], environmental factors [11], socio-psychological factors [12], and genetic factors [13] (Figure 1). The incidence of POF is about 1.0% globally, while in China, it is 1%–3.8%. Primary amenorrhea accounts for 20%–28% of POF cases, secondary amenorrhea accounts for about 4%–20% of cases, and about 74%–90% of POF cases have unknown etiology. The incidence of POF has been increasing in recent years with the development of the economy, changes in social relationships, and unhealthy lifestyles [14–16].

At present, the most common clinical treatment for POF is still hormone replacement therapy (HRT), but other therapies include in vitro activation, stem cell therapy, tissue engineering, and regenerative medicine. HRT is considered to reduce the risk of infection, osteoporosis, cardiovascular disease, and urogenital atrophy and improve the quality of life of women with POF. However, HRT does not fully restore ovarian function, and some studies have reported that HRT is a predisposing factor for breast cancer [17]. Therefore, clinicians are still looking for a new method to treat POF through complementary and alternative medicine (CAM). CAM is usually defined as “non-traditional” medicine according to the recommendations of the National Center for Comprehensive and Integrative Health (NCCIH). If unconventional methods or products are used together with conventional drugs, it is called complementary medicine, and if an unconventional method is used instead of standard treatment, it is considered an alternative method [18]. CAM includes many products and medical practices that are not conventional therapies in western countries, including not only traditional medicines and folk therapies, but also many new therapies that cannot be covered by medical insurance, such as traditional Chinese medicine (TCM; including Chinese herbal medicine, acupuncture, qigong, etc.), Indian medicine, medicinal food, health food, aromatherapy, vitamin therapy, dietary therapy, psychotherapy, spa therapy, and oxygen therapy [19, 20]. CAM is favored by many countries and nationalities because of its natural ingredients and methods, its convenience, and its low costs. It is also an effective strategy to alleviate the pain related to many diseases. Reports have suggested that the rate of CAM application has reached 9.8%–76.0% globally and that roughly 40% of adults use at least one type of CAM to treat a wide range of conditions in the USA [21, 22]. This article updates the progress in the research and application of CAM in the treatment of POF.

## 2. Single Herbal Medicines and Their Active Ingredients

Chinese herbal medicines have excellent efficacy in the treatment of POF, and many compound Chinese medicines have been widely used in the clinical treatment of POF due to their many advantages. Single herbal medicines are the basis for the research into compound Chinese medicines, and some of their active ingredients provide indications for the use of different Chinese herbal medicines in the treatment of POF. Current studies have found that the potential mechanisms of single herbal medicines and their active ingredients include estrogen-like effects, promoting DNA damage repair, enhancing anti-inflammatory and antioxidant capacity, regulating the expression of related pathways and proteins, and affecting prostaglandin biosynthesis, apoptosis, aging-associated, autophagy, etc., to delay POF.

### 2.1. Epimedium and Icariin

Epimedium, a representative of Chinese herbal medicines, has the ability to tonify the kidney and is commonly used to treat female infertility, irregular menstruation, amenorrhea, POF, and other diseases. One of the main active ingredients of Epimedium is icariin. Studies have shown that icariin has an obvious estrogen-like effect that can significantly increase the uterine coefficient, endometrial epithelial thickness, and serum E2 levels in ovariectomized mice [23]. In a rat model of POF, icariin could significantly increase the serum level of anti-Müllerian hormone (AMH), possibly by promoting the secretion of AMH in ovarian granulosa cells (GCs) and restoring normal follicular recruitment and maturation to maintain the ovarian reserve [24]. Li et al. found that icariin was effective in reducing ovarian damage by promoting DNA damage repair, suggesting that icariin might be used as a protective agent against POF [25].

### 2.2. Semen Cuscutae and TFSC/Cuscuta Flavonoids

Semen cuscutae is an important tonic for kidney yang and is commonly used in the treatment of gynecological diseases. Its main active chemical ingredient is Cuscuta flavonoids, which have significant effects on improving and enhancing the function of the human reproductive endocrine system. In a rat model of POF, total flavonoids from Semen cuscutae (TFSC) had a significant restorative effect on the estrous cycle and ovarian endocrine function and promoted follicular development and GCs proliferation in the ovary, indicating that they had estrogen-like effects [26]. Huang Changsheng believed that quercetin might be one of the main effective ingredients in Cuscuta flavonoids for the treatment of POF, and in a rat model of POF, both Cuscuta flavonoids and quercetin alone could inhibit the process of POF through activation of the phosphatidylinositol 3-kinase (PI3K)/protein kinase B (Akt) signaling pathway [27, 28].

### 2.3. Pueraria Lobata and Puerarin

The main active ingredients in Pueraria lobata are isoflavones and compound isoflavones. Puerarin is a 4,7-dihydroxy-8-*β*-D-glucosyl isoflavone and is the most important active ingredient of Pueraria lobata, and it has different degrees of estrogen-like effects [29]. Bcl-2-associated X protein (Bax) and B-cell lymphoma 2 (Bcl-2) play important roles in the anti-apoptotic effect in the Bcl-2 family, and Zhang et al. [30] found that puerarin could regulate the activity of Bax and Bcl-2 and inhibit apoptosis in ovarian tissue in a mouse model of POF and thus restore ovarian function. The expression of mouse vasa homolog (Mvh) and octamer-binding transcription factor 4 (OCT4) maintain the activity of female germline stem cells, and Chen et al. [31] found that puerarin not only activated the Wnt/*β*-catenin signaling pathway but also increased the expression of the antioxidant factors superoxide dismutase 2 (SOD2) and nuclear factor erythroid 2-related factor (Nrf2) to reduce oxidative stress.

### 2.4. Ginseng and Rg1

Ginseng is a traditional anti-aging drug, and its active ingredients are mainly composed of ginsenosides. The ginsenosides can be divided into three categories, namely ginseng diols (e.g., Rb1, Rb2, Rc, Rd, F2, etc.), ginseng triols (e.g., Re, Rg1, Rg2, Rf, Rh1, etc.), and pentacyclic triterpenoid saponins such as Ro [32]. The p16 and p53–p21–p19 pathways play an important role in the aging process, and Rg1 not only upregulates the expression of follicle-stimulating hormone receptor (FSHR) in the GCs of POF mice but also downregulates aging-associated proteins in the p19–p53–p21–p16 pathway and enhances the anti-aging capacity and fertility of POF mice by improving the anti-inflammatory and antioxidant capacity of the ovary [33]. Another experiment has shown that Rg1 effectively regulates the physiological status of the ovary, induces the expression of light-chain 3 (LC3)-II to increase autophagy levels, and may delay POF by activating the PI3K/Akt/mammalian target of rapamycin (mTOR) autophagy pathway [34].

### 2.5. Other Single Herbal Medicines

Hematopoietic prostaglandin D synthase (HPGDS), phospholipase A2-IVA (PLA2G4A), and prostaglandin-endoperoxide synthase 1 (PTGS1) are involved in prostaglandin biosynthesis in the body, and American ginseng affects the transformation of prostaglandin H2 (PGH2) into prostaglandin D2 (PGD2) by downregulating the expression of HPGDS and PTGS1 in the ovary and thus participates in the regulation of the reproductive system [35]. Animal models have shown that American ginseng plays a role in regulating prostaglandin biosynthesis, promoting ovulation, and preventing ovarian aging, which expands our understanding of the pharmacological activity of American ginseng as an anti-POF drug [36]. The expression of PLA2G4A is positively correlated with POF, while the expression levels of pregnancy-associated plasma protein-A, stanniocalcin-2, C-C motif chemokine ligand 2, and NEL-like protein 1 are negatively correlated with POF, and Ge et al. [37] confirmed in animal models that American ginseng can prevent and alleviate POF in rats by altering the expression levels of POF-related genes in ovarian tissues. These studies indicate that American ginseng is a potential clinical treatment for the prevention of POF.

The preparation made from Cistanche formulas can improve the clinical symptoms of menopausal syndrome, and follicle-promoting and luteinizing effects of Cistanche can regulate the endocrine function of female mice with kidney deficiency. Experiments have shown that Cistanche polysaccharide significantly improves the endocrine regulatory mechanisms of the body and has an inhibitory effect on POF by affecting the expression of tumor necrosis factor-alpha (TNF-*α*), interferon-gamma (IFN-*γ*), and the apoptosis-related protein Bcl-2/Bax [38, 39].

Angelica is an important gynecological medicine commonly used in Chinese herbal preparations, and Angelica polysaccharide is the main active ingredient. Animal experiments have found that Angelica polysaccharide can increase the activity of SOD and inhibit the level of malondialdehyde in the blood of mice with POF and that it promotes both oxidative stress and antioxidant capacity through the Akt/Forkhead box subgroup O3 (FOXO3) pathway, thus providing a novel approach for the treatment of immune-related POF [40].

Lycium barbarum polysaccharides are one of the main ingredients isolated from Lycium barbarum, a characteristic plant in Ningxia. These polysaccharides regulate endocrine production and maintain ovarian function in mice by slowing down ovarian damage caused by anti-zona pellucida antibody, possibly through both direct actions on immunoreactive cells and indirect actions on the hypothalamic pathway [41].

A study showed that high-dose maca powder could restore ovarian function and the abnormal estrous cycle, and improve the ovarian index and serum reproductive hormone levels of POF rats with kidney yang deficiency syndrome and that it has certain conservation effects on the ovary [42]. Oyster polypeptide plays an anti-oxidative role through the SIRT1-FOXO3a-SOD2 axis and protects against POF by reducing apoptosis [43]. The effectiveness of single herbal medicines and their active ingredients in the treatment of POF is summarized in Table 1.

## 3. Compound Chinese Medicines

Compound Chinese medicines are composed of two or more kinds of herbs that are boiled in water, and the residue is removed to obtain a clear liquid for Chinese medicine decoctions or is further processed into other dosage forms such as Chinese patent medicines, pills, powders, or creams [19]. Compound Chinese medicines have been used to treat diseases for thousands of years and have formed their own materia medica that is separate from traditional western medical practice. More and more studies have shown that compound Chinese medicines have overall advantages in the treatments of diseases due to their ability to simultaneously affect multiple targets and pathways, and this has attracted more and more attention in the treatment of POF compared with the efficacy and side effects of pharmaceutical drugs. Several studies have shown that compound Chinese medicines have a positive effect on POF, and the side effects are significantly less than for pharmaceutical drugs. Compounds extracted from Chinese herbal medicines can significantly reduce oxidative stress in the ovary and reduce apoptosis in ovarian GCs and oocytes. Thus, they play an important role in the treatment of POF by delaying apoptosis and regulating the secretory function of ovarian GCs and have significant advantages in increasing serum E2, reducing serum FSH levels, and improving clinical symptoms [44–47].

### 3.1. Chinese Medicine Decoctions

Chinese medicine decoctions, known in ancient times as “Tang Ye,” are important traditional preparations in TCM due to their ease of consumption, fast absorption, large drug load, and remarkable curative effect. The decoctions can be fully adapted to the needs of syndrome differentiation and treatment in TCM because of their flexibility, simplicity, low cost, quick effect, and the use of water as the solvent [48]. Chinese medicine decoctions that are commonly used in the clinical treatment of POF include Zuogui pill (ZGP), Bushen Huoxue decoction (BHD), Erxian decoction (EXD), and Yulin decoction.

#### 3.1.1. ZGP

ZGP, from Jingyue Quanshu, is a classic prescription for nourishing yin and tonifying the kidney and is widely used in the treatment of POF. According to TCM, women are kidney-based and POF is responsible for kidney deficiency. By nourishing yin and tonifying the kidney, filling the lean marrow, improving perimenopausal symptoms of POF, correcting sexual hormone disorders, and promoting the recovery of ovarian function, ZGP can not only improve the curative effects of western medicine but can also reduce side effects caused by hormone drugs without any serious adverse events [49–51]. Zeng et al. [52] showed that after ZGP treatment female rats showed an increase in ovarian volume, the ratio of total ovarian weight to body weight, and serum AMH and E2 levels and a decrease in serum FSH levels. Peng et al. [53] established a control group, model group, three ZGP groups (high-dose, medium-dose, and low-dose), and a triptorelin group to study ZGP's inhibition of mitochondrial-dependent apoptosis of follicles in POF rats. They found that ZGP inhibited follicle loss after exposure to chemotherapeutic drugs and improved the estrous cycle in rats. Further mechanistic studies showed that the protective effect of ZGP is related to the inhibition of the activation of the mitochondrial-dependent apoptosis cascade at the gene and protein levels. By inhibiting the expression of the pro-apoptotic molecule Bax and increasing the expression of the anti-apoptotic molecule Bcl-2, ZGP can reduce the level of serum FSH and increase the level of serum E2. It has also been shown that ZGP upregulates the protein expression of growth differentiation factor-9 and its signal transduction protein Smad2 in POF mouse ovaries, and thus ZGP can promote the recruitment of primordial follicles, promote follicular development, and inhibit follicular atresia [54].

#### 3.1.2. BHD

BHD [55–57] is a prescription developed by Professor Zhu Nansun, a master of Chinese medicine, and it exerts its therapeutic effects by tonifying the kidney and invigorating the blood, which benefits the kidney and fills the essence, fills the qi and blood, promotes blood circulation, and unblocks the collaterals to promote normal menstruation. Song et al. [58] verified the clinical efficacy of BHD in the treatment of POF patients by comparing the oral BHD group and the oral estradiol or estradiol dydrogesterone tablets group. Their results showed that BHD in the treatment of POF could significantly improve the TCM symptoms of patients—including hot flashes, night sweats, and other clinical manifestations—reduce the levels of serum FSH, mir-23a, and ovarian artery resistance index, and increase the level of AMH. Liu et al. [59] studied the effect of BHD on immune-related POF mice and found that compared with the model group, there was a significant increase in the number of mature ovarian follicles and a decrease in the number of atretic follicles in the high-dose group, medium-dose group, low-dose group, and estradiol valerate group of BHD, demonstrating that BHD can improve ovarian function by upregulating the protein expression of transforming growth factor-beta 1 (TGF-*β*1), transforming growth factor-beta receptor II (TGF-*β* RII), and Smad2/3 in GCs. BHD can promote normal levels of ovarian hormone secretion and promote the increase in mature follicles and the formation of primordial follicles and a large number of primary follicles through the upregulation of PI3K, Akt, and Bcl-2 protein expression in GCs [60].

#### 3.1.3. EXD

EXD is derived from the clinical manual of TCM formulations, and it warms the kidney, fills the essence, and reconciles the Chong Ren. In recent years, clinical observations and research on EXD in the treatment of POF have shown that the decoction has a clear effect on POF [61, 62]. Studies have shown that EXD has an effect on serum inflammatory factors and related growth factors in a rat model of POF. Compared with the low EXD dose group and the medium EXD dose group, the high-dose group showed significantly decreased serum levels of TNF-*α*, IFN-*γ*, FSH, and LH, significantly increased protein expression of vascular endothelial growth factor and basic fibroblastic growth factor in ovarian tissue, and increased levels of E2, showing that EXD could improve the level of sex hormone in a rat model of POF and promote the recovery of ovarian function [63]. In another study [64], treating POF mice with EXD restored the ovarian cycle to near or above the normal ovarian index, brought serum E2, FSH, and LH levels close to normal, the increased the numbers of CD3+ T-cells, CD4+ T-cells, and the CD4+ T-cell/CD8+ T-cell ratio, decreased the number of CD8+ T-cells, and increased the expression of BMP15 and Akt.

#### 3.1.4. Other TCM Decoctions

Based on the “liver and kidney theory” [65], Longjiang Han's Department of Gynecology applies Jiawei Yuyin decoction for tonifying the kidney and soothing the liver to provide symptomatic treatment for liver depression and kidney deficiency related to POF, and the patients' perimenopausal symptoms are significantly relieved and the serum levels of sex hormones return to normal. Modified mulberry decoction (MMD) has the effects of tonifying the liver and kidney, nourishing the blood and essence, and harmonizing Chong Ren. Wang et al. used estradiol valerate and cyproterone tablets as their control group and MMD as their treatment group. The results showed that the effective rate of the control group was 66.67% while that of the treatment group was 86.67%, and after treatment, the TCM syndrome scores and FSH and LH levels in the treatment group were lower than those in the control group and the E2 level was higher than in the control group. Their study showed that MMD could effectively improve the clinical symptoms of patients with POF, regulate the level of serum hormones, and promote menstrual regularity [66]. Modified Bazhen Decoction (MBD) [67] is effective in the treatment of POF. Professor Li [68] used the empirical formula “Yangshu Bazhen Decoction,” which was modified from the ancient formula “Bazhen decoction,” to treat POF by emphasizing the harmony of liver and kidney, paying attention to emotional treatment, balancing yin and yang, and regulating Chong Ren, which achieved good curative effects. In addition, Danggui Buxue decoction [69], Siwu decoction [70], Wenjing decoction [71], Bushen Jianpi formula [72], and other TCM decoctions have good effects in the treatment of POF, and these emphasize the flexible composition and good curative effect of TCM decoctions and fully demonstrate the theory of disease differentiation and treatment using TCM. The effect of TCM decoctions on POF is summarized in Table 2.

### 3.2. Chinese Patent Medicines

Chinese patent medicines use Chinese herbs as raw materials, and these are processed into a certain dosage form according to the specified prescription and preparation process. They have the characteristics of stable nature, definite curative effects, relatively weak side effects, and convenience of consumption, transport, and storage [73–75].

#### 3.2.1. Kuntai Capsule (KTC)

KTC is made according to the ancient prescription found in the Treatise on Febrile Diseases. It can effectively regulate women's endocrine levels, improve ovarian function, and prevent the decline of ovarian function. It can be used either alone or in combination with sex hormones to treat POF [76, 77]. Zhang et al. [78] found that KTC can regulate the estrous cycle, increase hormone secretion, improve fertility, and significantly reduce follicular atresia in the case of impaired ovarian function. Transmission electron microscopy showed that KTC could effectively maintain the ultrastructure of the mouse ovary, terminal deoxynucleotidyl transferase dUTP Nick end labeling (TUNEL) staining confirmed that KTC decreased apoptosis, and Western blot showed that KTC could reduce the expression of AMH, SOD2, Bcl-2, and Bax.

#### 3.2.2. Kunbao Pill (KBP)

KBP [79, 80] has the effects of restoring deficiency of qi and blood, weakness of kidney qi, and imbalance of yin and yang, nourishing the liver, kidney, and blood, calming the nerves, and dredging the collaterals, and it is widely used in the treatment of POF in the clinic. Li et al. explored the effects of KBP on the prevention and treatment of a rat model of POF and showed that the serum FSH, LH, and ovarian TGF-*β*1 levels were significantly decreased in the low-, medium-, and high-dose groups of KBP and combined estrogen group. They also found that serum E2 levels significantly increased and that stem cell factor expression levels significantly decreased in the medium- and high-dose KBP groups and combined estrogen group, and the connective tissue growth factor expression in ovarian tissue significantly decreased in the high-dose KBP group and combined estrogen group. Together, these results indicate that KBP has the effect of regulating the hormone levels of POF, which can reduce the expression of connective tissue growth factor, TGF-*β*1, and stem cell factor in ovarian tissues to relieve ovarian fibrosis damage and to promote the growth and development of early follicles and thus prevent the occurrence of POF [81].

#### 3.2.3. Other Chinese Patent Medicines

Chinese patent medicines can improve the clinical symptoms of POF and regulate the serum levels of hormones. Zishen Yutai pill (ZYP) has the effects of tonifying the kidney and spleen, nourishing blood, calming the fetus, supplementing qi, and nourishing yuan. It can effectively promote the blood supply to the female sexual organs and promote follicular development and progesterone secretion. The prescription has a good effect on promoting ovarian function. In one study, 78 patients with POF were randomly divided into a control group who took estradiol valerate tablets orally and an observation group who took estradiol valerate tablets combined with ZYP orally. The improvement in FSH, LH, and E2 contents in the observation group was significantly better than in the control group [82, 83]. Fuke Yangrong capsule is a compound preparation of TCM, and it has the effects of promoting blood circulation and menstruation, supplementing qi, nourishing the blood, tonifying the kidney, and soothing the liver. It can promote the development of the corpus luteum, accelerate the excretion of follicles, and improve ovarian function. Xiong treated patients using a sequential artificial cycle of estrogen and progesterone in the control group and a sequential artificial cycle of estrogen and progesterone combined with Fuke Yangrong capsule in the study group. The results showed that the levels of E2, FSH, and LH in the study group were significantly better than those in the control group, and this led to a significant increase in the number of sinus follicles and endometrial thickness and improved the level of sex hormones and the quality of sexual life, and thus is worthy of clinical promotion [84, 85]. Qilin pill has the functions of tonifying the kidney and essence, supplementing qi, and nourishing blood, and studies have shown that Qilin pill combined with estradiol valerate tablets can quickly and significantly reduce the serum levels of FSH and LH, increase the level of E2, and restore menstruation [86, 87].

### 3.3. Other Forms of Compound Chinese Medicine

Chinese medicine cream formulas are good at tonifying deficiencies. They are a commonly used TCM preparation in the gynecological clinic and are widely used because of their characteristics of slow onset of action and safety for long-term use, which is suitable for the diagnosis and treatment of POF. Moreover, the taste of Chinese medicine creams is better than Chinese medicine decoctions, which greatly improves the medication compliance of patients and thus is favored by doctors and patients [88]. To verify the efficacy of Bushen Tiaojing cream formula (BTCF) in the treatment of POF, Lu et al. [89] randomly divided 120 patients into a cream formula group, a Chinese medicine group, and a Western medicine group. In the cream formula group, the BTCF was prepared and decocted for oral administration. In the Chinese medicine group, self-prepared herbal medicine was used, and in the western medicine group, HRT was applied. After three courses of treatment, the results showed that the improvement of clinical symptoms in the cream formula group was better than that in the Western medicine group and Chinese medicine group. Compared with the Western medicine group, the cream formula group had clear advantages in treatment effect, the serum levels of E2 in the cream formula group and Chinese medicine group were higher than in the western medicine group, and the levels of FSH and LH were lower than in the western medicine group. BTCF has a significant clinical effect in the treatment of POF, and it improves clinical symptoms such as irregular menstruation, and it effectively regulates sex hormone levels and immune function [90, 91]. Yunkang oral solution (YKos) [92] has the effects of strengthening the spleen, nourishing the blood, and calming the fetus. A rat model of POF was prepared by giving cyclophosphamide. Compared with the model group, the serum E2 level of rats in the YKos group increased significantly, the FSH content decreased significantly, the ovarian and uterine coefficients increased significantly, the pathological changes of ovarian and uterine tissues improved significantly, and the expression of gonadotropin-releasing hormone receptor (GnRHR) and FSHR protein in the ovary increased significantly, indicating that YKos can effectively repair the damage to the reproductive system and can restore ovarian function through the regulation of the GnRHR-FSHR signaling pathway. The efficacy of Chinese patent medicines and other forms of compound Chinese medicines in the treatment of POF is summarized in Table 3. In addition, Ren et al. searched the Chinese science and technology journal database (VIP), the Wanfang Digital Journal Full-text Database, the China National Knowledge Infrastructure (CNKI), and other TCM literature on POF over the past 10 years and identified a total of 180 articles that met the inclusion criteria to summarize the Chinese herbal medicines with a high frequency of use in the treatment of POF as shown in Table 4 [93].

## 4. Acupuncture and Moxibustion

Acupuncture and moxibustion are widely used and have a variety of treatment forms. In addition to manual acupuncture and electroacupuncture stimulation, acupoint embedding and auricular acupoint pressure have also attracted much attention because of their simple operation and prolonged acupoint stimulation. Moxibustion combined with Chinese medicine decoctions can also achieve a remarkable therapeutic effect. Acupuncture and moxibustion therapy can adjust the balance of qi, blood, yin, and yang by stimulating acupoints. This has the characteristics of simple operation, safety, efficiency, and good efficacy and has been widely used in the treatment of POF. In addition, the combination of acupuncture and moxibustion with Chinese medicine and western medicine can have synergistic therapeutic effects, so such combinations are often used in clinical practice. In clinical treatment, the selection of acupoints is crucial for the therapeutic effect on the disease. Zhang et al. [94] summarized the commonly used therapeutic acupoints through a literature review of acupuncture treatments of POF, and this provides a useful reference for the clinical treatment of the disease (Table 5).

### 4.1. Acupuncture

In a rat model of POF, it was found that acupuncture regulated the expression levels of genes and proteins related to the PI3K/Akt/mTOR signaling pathway, promoted an increase in serum E2 level, and restored ovarian function [4, 95]. Clinical studies have shown that acupuncture can not only actively adjust ovarian status in the early stage of POF but can also improve the menstrual situation, perimenopausal symptoms, and serum sex hormone levels, increase clinical efficiency, and create better conditions for pregnancy [96, 97]. Yao et al. [98] needled the Guanyuan (RN4), Guilai (ST29), Taichong (LR3), Taixi (KI3), Xuehai (SP10), Sanyinjiao (SP6), Zigong (EX-CA1), Yinlingquan (SP9), Zusanli (ST36), Shuidao (ST28), Dahe (KI12), and Tianshu (ST25) acupoints prior to ovulation and needled the Ciliao (BL32), Shiqizhui (EX-B7), Ganshu (BL18), Shenshu (BL23), Geshu (BL17), and Pishu (BL20) acupoints after ovulation and compared the effects to HRT. The results showed that the total effective rate of the acupuncture group was 90.4% and the expression levels of IFN-*γ* and TNF-*α* decreased while the levels of LH, FSH, and E2 improved. The umbilical cord is an important orifice in the human body and is the hub of qi movement flow in the whole body. Professor Zhang Yongchen [99] developed the clinical treatment of acupuncture combined with umbilical cord therapy in the treatment of POF and used blood prick therapy to dredge the local qi and blood to treat both the symptoms and the root cause, and this had a significant curative effect and reduced patients' pain and side effects and thus is worthy of clinical promotion and application.

### 4.2. Moxibustion

Moxibustion therapy regulates the body's disordered physical and chemical functions by regulating the flow of qi and blood to prevent and treat disease [100]. Experiments in animal models showed that moxibustion of RN4 and SP6 can restore ovarian function and hormone levels, reduce the content of inflammatory factors IL-6 and IL-1*β*, and downregulate the expression levels of phosphorylated P-PI3K, P-Akt, and P-MTOR in ovarian tissues [101]. The toll-like receptor 4 (TLR4)/nuclear factor kappa B (NF-*κ*B) signaling pathway is the initial signal of inflammatory response. Moxibustion not only inhibits the TLR4/myeloid differentiation factor 88 (MyD88)/NF-*κ*B signaling pathway but also indirectly decreases nod-like receptor protein-3 (NLRP3), the precursor of IL1*β* (Pro-IL1*β*), and the precursor of IL18 (Pro-IL18). It can also directly inhibit pyroptosis induced by the thioredoxin-interacting protein (TXNIP)/NLRP3/Caspase1 signaling pathway and can regulate cell death through pyroptosis to alleviate ovarian failure in POF [102]. In addition, Liu [103] used Shenque moxibustion, Guanyuan moxibustion, and fire-dragon moxibustion to treat patients with POF and found that moxibustion improved patients' menstrual activity, clinical symptoms, and serum sex hormone levels and that it was easy to perform and accept and is a safe and effective method for the clinical treatment of POF.

### 4.3. Electroacupuncture Stimulation

Electroacupuncture stimulation of acupoints can effectively activate the functions of relevant organs. Through different intensities of electrical stimulation, it can not only increase the blood supply and nutrition of the treatment site and improve microcirculation but can also regulate neuroendocrine function [100, 104]. In a rat model of POF, it was found that electroacupuncture could improve the local morphology of the ovary, inhibit follicular atresia, promote follicular development, and improve ovarian function [105]. It protects the ovary by upregulating the expression of the apoptosis suppressor Bcl-2 protein and downregulating the expression of the pro-apoptotic factor Bax protein in ovarian GCs, and it improves POF by mediating the PI3K/AKT/mTOR pathway [106, 107]. Other animal model experiments have shown that electroacupuncture has a good therapeutic effect on POF, which is achieved by inhibiting ferroptosis and apoptosis that are induced by glutathione peroxidase 4 (GPX4) targeting the xC-system [108]. In addition, Zhang et al. found that warm acupuncture at “RN4” combined with electroacupuncture at “SP6” could regulate the serum sex hormone levels, improve the reproductive endocrine environment, and reduce the inflammatory response of the ovary in a rat model of POF [109].

### 4.4. Clinical Application of Combined Acupuncture and Moxibustion

Acupuncture and moxibustion therapy are often used in combination in clinical application. Wang et al. [110] used abdominal acupuncture combined with moxibustion to treat POF, and Yu et al. [111] used umbilical needle therapy combined with mixed moxibustion to treat POF. In addition, Wu et al. [112] randomly divided 50 patients with POF into an acupuncture group and a western medicine group. The acupuncture group used ST36 and RN4 warm acupuncture combined with Baliao (BL31, BL32, BL33, and BL34) ginger moxibustion, and the western medicine group was given oral climen. The results showed that in the acupuncture group, FSH and FSH/LH decreased, E2 increased, the peak systolic velocity of ovarian artery blood flow signal increased, the artery resistance index and pulsatility index decreased, the ovarian volume increased, and the AFC increased. The total effective rate was 92.0%, which was higher than that of the western medicine group (88%). In addition, Tian et al. [113] applied electroacupuncture combined with heat-sensitive moxibustion to treat 60 patients with POF, and its total effective rate reached 93.3% with the improved menstrual cycle and symptom scores.

### 4.5. Acupuncture and Moxibustion Combined with Drugs

Acupuncture is often used as an auxiliary treatment method in TCM and western medicine to adjust endocrine levels and improve the clinical symptoms and the pregnancy rate of infertility patients with POF [114–116]. Lai et al. [117] proposed the clinical use of “Tongyuan acupuncture” combined with TCM in the treatment of POF. Studies have found that moxibustion combined with artificial cycle therapy in the treatment of POF can adjust the levels of sex hormones and improve clinical indicators compared with the effect of artificial cycle therapy alone [118, 119]. In addition, Chi [120] used Yougui pills, acupuncture, and moxibustion combined with sequential therapy to treat POF, and the results showed that the effective rate was up to 90.48%, the TCM syndrome score and Kupperman score significantly reduced, and the ovarian function index, hemodynamic index, and sex hormone levels significantly improved. Acupuncture and moxibustion combined with Chinese and western medicine can not only reduce the incidence of adverse reactions and improve the safety of treatment but can also increase the clinical efficacy and is thus worth promoting [121–123]. Some studies have shown that electroacupuncture combined with compound Chinese medicines has good efficacy in the treatment of POF, but the sample sizes in the studies were small, and the mechanism of action and long-term efficacy need to be further observed and studied [124, 125].

### 4.6. Acupoint Catgut-Embedding

Acupoint catgut-embedding therapy is an improved acupuncture method in which biodegradable medical sutures are embedded into specific acupoints and regions of the body. This can stimulate the meridians and harmonize qi and blood and has the advantages of simple operation and long stimulation effect, and thus it has become important in the treatment of gynecological diseases and can be used for the treatment of POF with good efficacy [126, 127]. Chen et al. [128] used Chinese medicine for tonifying the kidney and nourishing the liver combined with acupoint catgut-embedding to treat POF, and the total effective rate of clinical efficacy reached 86.67% and significantly improved clinical symptoms such as menstrual cycle, vaginal dryness, and loss of sexual desire, and it increased serum sex hormone levels, endometrial thickness, and ovarian volume. In addition, studies on acupoint catgut-embedding combined with Chinese patent medicines, Chinese medicine decoctions, and western medicine have shown that acupoint catgut-embedding combination therapy can improve and restore ovarian function of patients, thus providing strong evidence for its clinical promotion [129–131].

### 4.7. Auricular Acupoint Pressure

Ear acupoints are closely related to the Zang-Fu organs and meridians, and stimulating specific acupoints of ear acupoints can regulate autonomic nerve function and relieve the uncomfortable symptoms caused by autonomic nerve dysfunction in patients with POF [132]. Shen [133] compared Modified Guishen Pill combined with auricular acupoint therapy (the combined treatment group) with sequential estrogen-progesterone therapy (the artificial cycle group) and observed the efficacy after 3 months of treatment. The results showed that the total effective rate of the combined treatment group was 93.3% and the TCM symptom score, FSH, and LH levels were significantly lower than those of the artificial cycle group, while the E2 level was significantly increased in the combined treatment group. Ye et al. [134] treated POF using Qingxin Jianpi decoction combined with auricular acupoint pressure, with a total clinical effective rate of 82.9% and proposed that regulating the heart and spleen is an important link that cannot be ignored in the treatment of POF. In conclusion, auricular acupoint pressure therapy is often used as an auxiliary therapy for the treatment of POF. Selecting auricular acupoints according to the results of TCM syndrome differentiation can not only enhance the pertinence of clinical treatment but can also reduce the adverse reactions of drug treatment and achieve better therapeutic effects.

## 5. Other Treatments

In clinical studies, psychotherapy, exercise therapy, oral vitamins, massage, and other methods have been shown to have good therapeutic effects in the treatment of gynecological diseases. These methods are often used in combination with hormones and Chinese herbal medicines, which can improve the therapeutic effect and the quality of life of patients.

### 5.1. Psychotherapy

POF causes a great deal of physical and psychological stress in women, so psychological nursing is essential in the treatment of this disease. Psychological suggestion, targeted care, strengthening communication with patients about the disease, and enhancing communication with family members [135, 136] are commonly used in the treatment of POF and can improve anxiety, depression, and quality of life and can increase treatment compliance and treatment effect in patients with POF [137]. Cui et al. [138] proposed a psychosomatic treatment with TCM for POF that is based on regulating the movement of qi. Clinical studies have shown that combination therapy such as the psychosomatic treatment of TCM and estrogen-progesterone combined with psychological counseling has clinical promotion and application value by improving the happiness index of patients with good clinical efficacy [139–143].

### 5.2. Exercise

There is a close causal relationship between exercise and human physical and mental health. Physical exercise can improve body functions, and regular exercise can reduce stress, improve negative moods such as anxiety and depression, support sleep, and reduce chronic stress-related diseases [144]. Animal experiments have also shown that exercise can improve depression-like behavior in ovariectomized rats [145]. In a clinical study, Wu et al. [146] found that Baduan Jin exercises improved ovarian function, increased ovulation rates, and improved the quality of life of patients with low ovarian reserve function. Exercise therapy is simple, easy to implement, and does not increase the patient's financial burden, and it has a high acceptance among patients and strong operability, which make it highly applicable to patients with POF [147].

### 5.3. Vitamins

Vitamin E is a fat-soluble vitamin with strong antioxidant effects. Reasonable supplementation of vitamin E can enhance the antioxidant protection of the ovary and can increase ovarian reserve. Vitamin E combined with HRT is often used in the clinical treatment of POF [148, 149]. Zou et al. [150] further suggested that coenzyme Q10 combined with vitamin E can enhance the protective antioxidant effect on the ovaries in elderly women, improve ovarian reserve, and increase ovarian responsiveness. It has been shown that POF is a high-risk factor for osteoporosis, and the combination of calcium tablets, calcitriol, and vitamin D has definite efficacy in the treatment of POF with osteoporosis [151].

### 5.4. Massage

Massage, which can relax tendons, invigorate blood, improve fitness, and prevent disease, is often used clinically in combination with Chinese herbal medicine in patients with POF. Such combined therapy can improve the levels of various serum sex hormones and has good efficacy in the treatment of POF [152, 153]. In addition, Feng et al. [154] adopted electroacupuncture combined with pelvic floor muscle massage, which can not only improve the local blood flow of the ovary but can also adjust the clinical symptoms and endocrine levels of the patients as a whole to treat POF.

### 5.5. Diet

TCM has always held to the concept of the homology between medicine and food. Studies have shown that a high-calorie diet may contribute to metabolic disorders including diabetes, obesity, and hyperlipidemia and may also affect female fertility by directly impairing oocyte health and differentiation or by indirectly interfering with the pituitary-hypothalamic axis [155]. Chen et al. [156] explored the relationship between dietary nutrition and POF by comparing different daily intakes of protein, carbohydrate, and dietary fiber in two groups of POF patients, and they proposed the view that a deficiency of carbohydrate and dietary fiber is associated with POF. However, there is still a lack of studies examining the relationship between dietary nutrition and POF, which needs to be explored further.

## 6. Conclusions

In recent years, clinical and scientific researchers have paid more attention to POF and its associated symptoms such as amenorrhea and infertility. As the research has progressed, more and more CAM therapies have become widely accepted and well used, including herbal medicine, acupuncture, psychology, exercise, vitamins, massage, diet, etc. These therapies can significantly improve the patient's symptoms and hormone levels and can be used in combination with other treatments to enhance their efficacy. However, to increase the benefits of these alternative medical interventions for POF patients worldwide, the standardization of effective CAM treatments, larger sample sizes, and more randomized controlled trials are still needed to confirm the effectiveness and safety of CAM for POF.

## Figures and Tables

**Figure 1:** Risk factors and etiology of POF.

**Table 1:** Summary of the curative effects of single herbal medicines in POF.

Single herbal medicine	Active ingredients	Outcomes	References
Epimedium	Icariin	FSH, LH↓; E2, AMH↑.	[24, 25]
Semen cuscutae	TFSC/cuscuta flavonoids	TFSC processing: E2↑. Cuscuta flavonoids processing: FSH↓; E2, AMH↑.	[26, 27]
Pueraria lobata	Puerarin	FSH↓; E2, AMH↑; Bcl-2↑; Bax, cleaved caspase-3↓; *β*-catenin, SOD2, Nrf2↑.	[30, 31]
Ginseng	Rg1	FSH↓; E2, AMH↑; IL-1b, IL-6, TNF-*α*↓; aging-associated proteins in the p19-p53-p21-p16 pathway↓, LC3-II↑.	[33, 34]
American ginseng	/	FSH↓; E2↑; HPGDS, PLA2G4A, PTGS1↓; PAPPA, STC2, CCL2, NELL1↑.	[34–37]
Cistanche	/	FSH↓; E2, AMH↑; IFN-*γ* and TNF-*α*↓; Bcl-2↑; Bax↓; Bcl-2/Bax ratio↑.	[39]
Angelica	AP	SOD↑; MDA↓; IL-1*β*, IL-6↓.	[40]
Lycium barbarum	LBP	FSH↓; E2↑; serum anti-zona pellucida antibody↓.	[41]
Maca	/	FSH, LH↓; E2↑.	[42]
Oyster	Oyster polypeptide	FSH↓; P↑; P53, Bad↓.	[43]

TFSC: total flavonoids from Semen cuscutae; AP: Angelica polysaccharide; LBP: Lycium barbarum polysaccharides. FSH: follicle-stimulating hormone; LH: luteinizing hormone; E2: estradiol; AMH: anti-Mullerian hormone; Bcl-2: B-cell lymphoma 2; Bax: Bcl-2-associated X protein; SOD2: superoxide dismutase 2; Nrf2: nuclear factor erythroid 2-related factor; IL-1b: interleukin-1b; IL-6: interleukin-6; TNF-*α*: tumor necrosis factor-alpha; LC3-II: light-chain 3 (LC3)-II; HPGDS: hematopoietic prostaglandin D synthase; PLA2G4A: phospholipase A2-IVA; PTGS1: prostaglandin-endoperoxide synthase 1; PAPPA: pregnancy-associated plasma protein A; STC2: stanniocalcin-2; CCL2 : C-C motif chemokine ligand 2; NELL1: NEL-like protein 1; IFN-*γ*: interferon-gamma; SOD: superoxide dismutase; MDA: malondialdehyde; IL-1*β*: interleukin-1beta.

**Table 2:** Summary of the curative effects of TCM decoctions on POF.

Chinese medicine decoction	Ingredients	Sample size	Interventions	Model used	Outcomes	References
Zuogui pill (ZGP)	Rehmanniae radix praeparata, cornel, yam, semen cuscutae, Chinese wolfberry fruit, radix achyranthis bidentatae, colla carapacis et plastri testudinis, and antler gelatin	*N* = 114	Control group, model group, low-ZGP group, high-ZGP group, low-dose estradiol valerate, high-dose estradiol valerate, DAPT group, and DAPT + low-ZGP group	SD rats	FSH↓; E2, AMH↑; ovarian volume↑; ratio of total ovary weight to body weight↑.	[52]

Bushen huoxue decoction (BHD)	Panax notoginseng powder, rhizoma cyperi, licorice, spatholobus suberectus stem, psoralea corylifolia, rhizoma curculiginis, semen cuscutae, cornel, angelica, epimedium, salvia miltiorrhiza, ligusticum wallichii, codonopsis pilosula, rehmanniae radix praeparata, and radix paeoniae alba.	*N* = 73	BHD group and western medicine group (estradiol or estradiol didroxyprogesterone tablets)	Human study	FSH↓; AMH↑; TCM syndrome score↓; mir-23a, ovarian artery RI↓.	[58]

Erxian decoction (EXD)	Rhizoma curculiginis, epimedium, morinda officinalis, anemarrhena, phellodendron amurense, and angelica.	*N* = 60	Normal group, model group, bujiale group, low-EXD group, medium-EXD group, and high-EXD group	SD rats	FSH, LH↓; E2↑; TNF-*α*, IFN-*γ*↓; VEGF, bFGF↑.	[63]

Modified mulberry decoction (MMD)	Fructus mori, lilium brownii, angelica, rehmanniae radix praeparata, radix paeoniae alba, epimedium, cistanche, and licorice.	*N* = 60	Control group: climen tablets treatment group: MMD	Human study	FSH, LH↓; E2↑; TCM syndrome score↓.	[66]

Modified bazhen decoction (MBD)	Bupleurum, angelica, ligusticum wallichii, radix paeoniae alba, glutinous rehmannia, codonopsis pilosula, atractylodes, poria cocos, licorice, antlers, radix achyranthis bidentatae, and rhizoma cyperi	*N* = 24	Control group, POF group, MBD group, and FES group	SD rats	XIAP↑; mir-23a, mir-27a↓.	[67]

Danggui buxue decoction (DBD)	Angelica and astragalus mongholicus	*N* = 50	Control group, model group, DBD group, quercetin group, and kaempferol group	SD rats	FSH, LH↓; E2, AMH↑; cytochrome c, Bax, p53 and IL6↓; ,ESR1, AR, Bcl-2↑.	[69]

Si-Wu-Tang (SWT)	Rehmanniae radix praeparata, angelica, paeonia lactiflora pall, and ligusticum wallichii	*N* = 36	Control group, model group, low-SWT group, medium-SWT group, high-SWT group, and DHEA group	Six C57BLmice	FSH, LH↓; E2, AMH↑; TCM syndrome score↓.	[70]

Wenjing decoction (WJD)	Evodia rutaecarpa, cassia twig, radix paeoniae alba, angelica, ligusticum wallichii, donkey-hide gelatin, ophiopogon japonicus, ginger, rhizoma pinelliae, moutan bark, ginseng, and licorice	*N* = 119	Control group: HRT (progynat + progesterone capsules) observation group: HRT (progynat + progesterone capsules), WJD, and acupuncture	Human study	FSH, LH↓; E2, AMH↑; TCM syndrome score↓.	[71]

DAPT: dual antiplatelet therapy; FES: Fufang Ejiao Syrup; DHEA: dehydroepiandrosterone; FSH: follicle-stimulating hormone; LH: luteinizing hormone; E2: estrogen; AMH: anti-Müllerian hormone; RI: resistance index; TNF-*α*: tumor necrosis factor-alpha; IFN-*γ*: interferon-gamma; VEGF: vascular endothelial growth factor; bFGF: basic fibroblastic growth factor; XIAP: X-linked inhibitor of apoptosis protein; IL6: interleukin-6; ESR1: estrogen receptor 1; AR: androgen receptor.

**Table 3:** Summary of the efficacy of Chinese patent medicines on POF.

Chinese patent medicine	Ingredients	Sample size	Interventions	Model used	Outcomes	References
Kuntai capsule (KTC)	Rehmanniae radix praeparata, rhizoma coptidis, donkey-hide gelatin, radix paeonia alba, poria cocos, and radix scutellariae.	/	/	/	FSH, LH↓; E2, AMH↑; Kupperman score↓.	[77]

Kunbao pills (KBP)	Fructus ligustri lucidi, raspberry, semen cuscutae, Chinese wolfberry fruit, fleeceflower root, tortoise shell, Chinese wolfberry root bark, adenophora tetraphylla, ophiopogon japonicus, wild jujube kernel, glutinous rehmannia, radix paeoniae alba, radix paeoniae rubra, angelica, spatholobus suberectus stem, nacre mother of pearl, dendrobium nobile, chrysanthemum, eclipta, folium mori, radix cynanchi atrati, anemarrhena, and radix scutellariae.	*N* = 60	Blank group, model group, low-KBP group, medium-KBP group, high-KBP group, and estrogen combination group	SD rats	FSH, LH↓; E2↑; TGF-*β*1↓; SCF↓.	[81]

Zishen yutai pill (ZYP)	Semen cuscutae, fructus amomi, rehmanniae radix praeparata, ginseng, parasitic loranthus, donkey-hide gelatin, fleeceflower root, folium artemisiae argyi, morinda officinalis, bighead atractylodes rhizome, codonopsis pilosula, cornu cervi degelatinatum, Chinese wolfberry fruit, teasel root, eucommia ulmoides	*N* = 80	The control group (estradiol valerate tablets), the observation group (estradiol valerate tablets combined with ZYP)	Human study	FSH, LH↓; E2↑; Kupperman score↓.	[82]

Fuke yangrong capsule (FYC)	Angelica, bighead atractylodes rhizome, rehmanniae radix praeparata, ligusticum wallichii, radix paeoniae alba, rhizome cyperi, motherwort, astragalus mongholicus, eucommia ulmoides, folium artemisiae argyi, ophiopogon japonicus, donkey-hide gelatin, licorice, dried tangerine peel, poria cocos, fructus amomi	*N* = 80	The control group (sequential artificial cycle of estrogen and progesterone) and the observation group (sequential artificial cycle of estrogen and progesterone combined with FYC)	Human study	FSH, LH↓; E2↑; TCM syndrome score↓.	[85]

Qilin pill (QLP)	Prepared fleeceflower root, eclipta, epimedium, semen cuscutae, cynomorium songaricum, codonopsis pilosula, radix curcumae, raspberry, Chinese wolfberry fruit, yam, red-rooted salvia root, astragalus mongholicus, radix paeoniae alba, pericarpium citri reticulatae viride, and fructus mori	*N* = 72	Climen tablet group and climen tablets combined with QLP group	Human study	FSH, LH↓; E2↑.	[87]

Bushen Tiaojing cream formula (BTCF)	Rehmanniae radix praeparata, yam, cornel, chinese wolfberry fruit, semen cuscutae, angelica, radix cyathulae, donkey-hide gelatin, motherwort, poria cocos, and moutan bark	*N* = 110	The control group (HRT) and the observation group (HRT combined with BTCF)	Human study	FSH, LH↓; E2↑; GDF-9, BMP-15↑.	[90]

Yunkang oral solution (YKos)	Yam, teasel root, astragalus mongholicus, angelica, rhizoma cibotii, semen cuscutae, parasitic loranthus, eucommia ulmoides, psoralea corylifolia, codonopsis pilosula, poria cocos, bighead atractylodes rhizome, donkey-hide gelatin, glutinous rehmannia, cornel, Chinese wolfberry fruit, smoked plum, radix paeoniae alba, fructus amomi, alpinia oxyphylla, radix boehmeriae, radix scutellariae, and folium artemisiae argyi	*N* = 108	Control group, CTX model group, positive control group and high-YKos, medium-YKos and low-YKos groups	SD rats	FSH↓; E2↑; ovarian coefficient, uterine coefficient↑; GnRHR, FSHR↑.	[92]

CTX: cyclophosphamide; FSH: follicle-stimulating hormone; LH: luteinizing hormone; E2: estrogen; AMH: anti-Müllerian hormone; TGF-*β*1: transforming growth factor beta1; SCF: stem cell factor; GDF-9: growth differentiation factor 9; BMP15: bone morphogenetic protein 15; GnRHR: gonadotropin-releasing hormone receptor; FSHR: follicle-stimulating hormone receptor.

**Table 4:** The frequency of use of Chinese herbal medicines for the treatment of POF.

Drug efficacy	Number	Percentage (%)	Chinese herbal medicines and frequency
Tonic drug	21	67.86	Rehmanniae radix praeparata 164, angelica 164, semen cuscutae 163, yam 109, Chinese wolfberry fruit 106, radix paeoniae alba 76, licorice 67, fructus ligustri lucidi 66, epimedium 87, eucommia ulmoides 54, dried human placenta 46, morinda officinalis 43, bighead atractylodes rhizome 38, antler gelatin 38, radix glehniae 13, fructus mori 13, donkey hide gelatin 11, amethyst 10, ginseng 10, radix pseudostellariae 9, ophiopogon japonicus 9
Drug for promoting blood circulation and removing stasis	11	11.77	Salvia miltiorrhiza 57, ligusticum wallichii 50, radix achyranthis bidentatae 28, radix cyathulae 24, safflower carthamus 24, spatholobus suberectus stem 23, motherwort 20, peach kernel 19, eupatorium 16, radix curcumae 10, motherwort fruit 10
Astringent drug	3	6.30	Cornus officinalis 110, raspberry 24, schisandra chinensis 17
Antipyretic drug	5	5.09	Moutan bark 39, phellodendron amurense 22, anemarrhena 21, rehmannia glutinosa 20, radix paeoniae rubra 20
Diuretic and hygroscopic drug	2	3.38	Poria cocos 67, alisma orientalis 14
Qi regulating drug	2	2.84	Rhizoma cyperi 48, dried tangerine peel 20
Drug for treating external syndromes	1	1.59	Bupleurum 38
Interior-warming drug	2	1.17	Cinnamomum cassia 17, radix aconiti carmichaeli 11

**Table 5:** Modern acupuncture selection for the treatment of POF.

Acupoint	International code	Meridians	Frequency of use	Percentage (%)
Guanyuan	RN4	Ren	34	73.91
Shenshu	BL23	Bladder	29	63.04
Sanyinjiao	SP6	Spleen	28	60.87
Zhongji	RN3	Ren	21	45.65
Zusanli	ST36	Stomach	19	41.30
Zigong	EX-CA1	Extra points	18	39.13
Pishu	BL20	Bladder	18	39.13
Taixi	KI3	Kidney	17	36.96
Taichong	LR3	Liver	16	34.78
Ganshu	BL18	Bladder	16	34.78
Xuehai	SP10	Spleen	15	32.61
Qihai	RN6	Ren	14	30.43
Guilai	ST29	Stomach	9	19.57
Dahe	KI12	Kidney	7	15.22
Ciliao	BL32	Bladder	7	15.22

## Data Availability

No data were used to support the findings of this study.
